The article "Shen-Ling-Bai-Zhu-San Enhances the Antipneumonia Effect of Cefixime in Children by Ameliorating Gut Microflora, Inflammation, and Immune Response" was retracted in 2023. Reasons: signs of a paper mill; suspected computer-generated content; unreliable results or conclusions; concerns about the data.

# Shen-Ling-Bai-Zhu-San Enhances the Antipneumonia Effect of Cefixime in Children by Ameliorating Gut Microflora, Inflammation, and Immune Response

**DOI:** 10.1155/2022/7752426

**Published:** 2022-09-07

**Authors:** Jinli Feng, Cheng Zhang, Houjun Chen, Ziliang Chen, Yongfeng Chen, Degen He, Qianyi Pan, Yongmao Zhou, Zhaoyang Chen, Xiaozheng Zhuang

**Affiliations:** ^1^Emergency Department, Zhongshan Hospital, Guangzhou University of Chinese Medicine, Zhongshan, Guangdong 528401, China; ^2^Clinical Laboratory, Zhongshan Hospital, Guangzhou University of Chinese Medicine, Zhongshan, Guangdong 528401, China; ^3^Pediatrics, Zhongshan Hospital, Guangzhou University of Chinese Medicine, Zhongshan, Guangdong 528401, China; ^4^Prevention and Health Section, Zhongshan Hospital, Guangzhou University of Chinese Medicine, Zhongshan, Guangdong 528401, China

## Abstract

**Objective:**

Shen-Ling-Bai-Zhu-San (SLBZS) is used for treating gastrointestinal disorders. However, the role of SLBZS in treating pneumonia in children is still unclear.

**Methods:**

In this study, children (≥2 and <9 years) with pneumonia were treated with 0.1 g cefixime (cefixime group) or 0.1 g cefixime + 9 g SLBZS (SLBZS + cefixime). The drugs were administered twice daily for 10 days. The therapeutic effects of the two groups were compared. The white blood cell (WBC), neutrophil, and lymphocyte counts; neutrophil-lymphocyte ratio (NLR); serum inflammatory factor levels; and gut microflora were assessed.

**Results:**

The clinical efficacy of SLBZS + cefixime treatment of pneumonia in children was higher than that of cefixime alone (93.3% *vs.* 86.7%). Both cefixime and SLBZS + cefixime treatments decreased the area of pulmonary inflammatory lesions, reduced white blood cell and neutrophil counts, neutrophil-lymphocyte ratio, inflammation, and increased lymphocyte count in children with pneumonia compared with those before treatment. Moreover, SLBZS enhanced the anti-inflammation and immunity-enhancing effects of cefixime in children with pneumonia. SLBZS + cefixime treatment decreased *Enterobacter*, *Enterococcus*, *Bacteroides*, and *Fusobacterium* counts and increased *Bifidobacterium* and *Lactobacillus* counts. Compared with the cefixime treatment group, the count of the six bacterial strains in the SLBZS + cefixime treatment group was closer to the normal level.

**Conclusion:**

SLBZS enhanced the antipneumonia effect of cefixime in children with pneumonia by ameliorating gut microflora, inflammation, and immune response.

## 1. Introduction

Pneumonia is a pulmonary infection caused by microbes such as bacteria, viruses, or fungi. This disease is commonly seen in infants, school-aged children, and adolescents and may occur throughout the year, with a high incidence rate during winter and spring [1, 2]. Pneumonia induces not only respiratory tract symptoms but also intrapulmonary complications and extrapulmonary systemic impairment, severely reducing the quality of life [3]. The therapeutic effect of the current treatments is not very satisfactory [4]. Thus, there is an urgent need to find alternative treatments to improve the current therapeutic strategies.

The article "Shen-Ling-Bai-Zhu-San Enhances the Antipneumonia Effect of Cefixime in Children by Ameliorating Gut Microflora, Inflammation, and Immune Response" was retracted in 2023. Reasons: signs of a paper mill; suspected computer-generated content; unreliable results or conclusions; concerns about the data.

Shen-Ling-Bai-Zhu-San (SLBZS), a traditional Chinese medicine prescribed for spleen deficiency (a traditional Chinese medicine syndrome type), was first used to treat diarrhea and loss of appetite and was proposed as a treatment in “Tai Ping Hui Min He Ji Ju Fang” in the Song Dynasty [5]. SLBZS has been extensively used to treat several diseases owing to its significant health-improving effects, such as enhancing blood sugar control and *β*-cell function, protecting from ulcerative colitis, and preventing inflammation and nonalcoholic steatohepatitis-induced liver injury [6, 7]. Moreover, SLBZS can suppress colitis-associated colorectal cancer by inhibiting epithelial-mesenchymal transition and myeloid-derived suppressor infiltration [8]. In addition, SLBZS has been shown to alleviate functional dyspepsia in rats and modulate the composition of gut microflora [9]. The distribution of gut microflora is closely associated with pneumonia; for example, neonatal gut microflora can regulate lung immunity to prevent pneumonia [10]. Moreover, gut bacteria, such as *Bifidobacterium* and *Escherichia coli*, were altered in children with recurrent pneumonia [11]. The gut microbiota enhances alveolar macrophage function to reduce inflammation during pneumococcal pneumonia infection [12]. A previous study found that SLBZS could be used to treat pneumonia, possibly by enriching the beneficial intestinal microbiota [13]. Our previous study revealed that SLBZS improved lung injury by regulating gut microbiota in the pneumonia mice model [14].

Cefixime has broad-spectrum activity against Gram pathogens and is used to treat pneumonia [15]. However, it remains unclear whether SLBZS can enhance the antipneumonia effect of cefixime in children. Therefore, we investigated the clinical therapeutic effect and the regulation of inflammation and gut microbiota of cefixime combined with SLBZS in children with pneumonia.

## 2. Materials and Methods

### 2.1. SLBZS Decoction

SLBZS was purchased from Tongrentang (SFDA approval number: Z1102O755; Beijing, China). Its composition is as reported in our previous study [14]. SLBZS (9 g) was dissolved in 100 mL of water.

### 2.2. Subjects

This randomized controlled study was conducted between January 2019 and June 2020 in the Emergency Department at Zhongshan Hospital, Guangzhou University of Chinese Medicine. A total of 60 children with pneumonia were enrolled. Pneumonia was diagnosed based on the guidelines for diagnosis and treatment of community-acquired pneumonia, acute onset, presence of cough and expectoration, rales in lung auscultates and lung shadows observed using laboratory examination, and considerably increased white blood cell (WBC) and neutrophil counts. Informed consent was obtained from the children's guardians. The study protocol was approved by the Ethics Committee of Zhongshan Hospital, Guangzhou University of Chinese Medicine (approval no.: 2017ZSZY-LLK-02). All methods were carried out in accordance with relevant guidelines and regulations. Consent to publish these details has been obtained from all individuals. All relevant personal information was hidden in the X-ray images. This experiment was performed in accordance with the Declaration of Helsinki ethical guidelines for clinical research.

The article "Shen-Ling-Bai-Zhu-San Enhances the Antipneumonia Effect of Cefixime in Children by Ameliorating Gut Microflora, Inflammation, and Immune Response" was retracted in 2023. Reasons: signs of a paper mill; suspected computer-generated content; unreliable results or conclusions; concerns about the data.

### 2.3. Inclusion Criteria

Children meeting the following criteria were included in the study: boys and girls aged ≥2 and <9 years, a diagnosis consistent with the criteria for pneumonia in children, no serious genetic, heart, liver, kidney, or other important organ diseases or dysfunctions, and not receiving antibiotics, biological agents, or drugs that regulate intestinal flora within a week before treatment.

### 2.4. Exclusion Criteria

Children were excluded from the study if they were seriously ill and needed hospitalization, were allergic to the drugs used in clinical observation, had a preexisting gastrointestinal disease or developed a gastrointestinal disease in the week prior to commencement of the study, and showed poor compliance, i.e., refused oral medicine or traditional Chinese medicines.

### 2.5. Study Design

For sample size calculations, 10 patients in each group were included in the preliminary experiment. The course of the disease was 15.3 ± 3.945 days in the cefixime group and 12.4 ± 2.716 days in the cefixime + SLBZS group. The disease' course was considered a comparative parameter for sample size estimation. The power of 80% (1-*β*) was obtained on both sides under an *α* = 0.05 test level. The mean comparison method was used to calculate the sample size. It was estimated that at least 46 subjects (power = 0.8106) were required. A total of 56 subjects (28 in each group) needed to be included in this study, assuming a 20% dropout rate. The above sample size estimation was carried out using PASS 15.0 software (NCSS, LLC, and Kaysville, UT, USA). Finally, the number of subjects per group was rounded to 30. In the present study, 60 children with pneumonia were randomly divided into the cefixime + SLBZS and cefixime groups at a 1 : 1 ratio. Random numbers assigned to each group were written on a piece of paper, placed in a sealed, opaque envelope, and given to the participants. The evaluators in the trial were unaware of the random assignment of the participants. The statistics and analysis of the data were completed by statisticians with no knowledge of grouping. Both groups were treated with antitussives and expectorants. The cefixime group received 0.1 g cefixime granules (Product ID: 2170104; SFDA approval number: H10940128; Baiyunshan Pharmaceutical General Factory, Guangzhou, China) dissolved in 100 mL of distilled water and administered once in the morning (8 : 00 AM) and evening (8 : 00 PM). The cefixime + SLBZS group received 9 g SLBZS and 0.1 g cefixime granules dissolved in 100 mL of distilled water, administered once in the morning (8 : 00 AM) and evening (8 : 00 PM) for 10 days. Clinical manifestations after treatment were used to evaluate whether the treatment was completed. Blood samples for routine blood tests and cytokine analysis and fresh fecal samples for gut microbiota analysis were collected before and after treatment. Additionally, chest radiographs of the two groups were analyzed before and after treatment.

The article "Shen-Ling-Bai-Zhu-San Enhances the Antipneumonia Effect of Cefixime in Children by Ameliorating Gut Microflora, Inflammation, and Immune Response" was retracted in 2023. Reasons: signs of a paper mill; suspected computer-generated content; unreliable results or conclusions; concerns about the data.

### 2.6. Observation Index

The therapeutic effects, chest X-ray results, and disease course of the two groups were compared before and after treatment to evaluate the efficacy of cefixime and SLBZS in treating pneumonia in children. For evaluation, the curative effect was divided into obviously effective, effective, and invalid effects. The obviously effective class had the following characteristics: a significantly reduced or absent cough; significantly reduced or absent lung rales; and the lungs that had returned to normal or with most lesions absorbed on X-ray examination. The effective class comprised the following characteristics: normal body temperature, less coughing, fewer rales in the lungs, and fewer lesions absorbed on X-ray examination. The invalid effects class consisted of the following characteristics: symptoms not significantly improved, lung rales not significantly reduced, and lesions not absorbed on X-ray examination. The following equation gives the total efficacy rate of the treatments:

(1) $$\begin{array}{c} \text{Total efficacy rate}=\frac{\left(\text{obviously effective}+\text{effective}\right)}{\text{total cases}}\times 100\%. \end{array}$$

### 2.7. Laboratory Test

WBC, neutrophil, and lymphocyte counts, as well as NLRs in patients before and after treatment, were detected using a BC-6800 automatic blood cell analyzer (Mindray Medical, Shenzhen, China). The C-reactive protein (CRP, bsk11041, Bioss, Beijing, China), procalcitonin (PCT, OKEH02858, Aviva Systems Biology, Beijing, China), interferon (IFN)-*γ* (bsk11013, Bioss), tumor necrosis factor (TNF)-*α* (bsk11014, Bioss), interleukin (IL)-1*β* (bsk11001, Bioss), IL-6 (bsk11007, Bioss), IL-8 (bsk11008, Bioss), and IL-10 (bsk11010, Bioss) levels in serum of patients before and after treatment were measured using enzyme-linked immunosorbent assay (ELISA). Finally, adverse reactions, including diarrhea, nausea, aches, rashes, dizziness, and abnormal liver and kidney function, were evaluated by an independent research assistant who was not involved in the screening or evaluation of the participants.

The article "Shen-Ling-Bai-Zhu-San Enhances the Antipneumonia Effect of Cefixime in Children by Ameliorating Gut Microflora, Inflammation, and Immune Response" was retracted in 2023. Reasons: signs of a paper mill; suspected computer-generated content; unreliable results or conclusions; concerns about the data.

### 2.8. Gut Microbiota Analysis

Fresh feces (>30 min) were collected, and a 1 g sample was placed in a sterile test tube with phosphate-buffered saline (PBS; 0.9 mL). Stool DNA from fresh feces was extracted via the E.Z.N.A.® Stool DNA Kit (Omega, Norcross, GA, USA), and DNA concentration was determined using a NanoPhotometer™ (Uvikon 923, USA). The numbers of *Enterobacter*, *Enterococcus*, *Bacteroides*, *Bifidobacterium*, *Lactobacillus*, and *Fusobacterium* were quantified by qPCR. Thereafter, stool DNA from each species and their standard plasmids were quantified by qPCR using a 7500 Fast Real-Time PCR System (Applied Biosystems, Waltham, MA, USA). The primer sequences were purchased from Sangon (Shanghai, China). The number of colony-forming units (CFUs) was counted and expressed as wet weight log_10_ CFU/g.

### 2.9. Statistical Analysis

Statistical analysis was performed using SPSS 19.0 statistical software (SPSS Inc., Chicago, IL, USA). Normally distributed data were expressed as means ± standard deviations and analyzed using Student's *t*-test between the two groups. A one-way analysis of variance was used for comparing multiple groups, followed by Tukey's post hoc test. Abnormally distributed data were expressed as the median (interquartile range) and analyzed using nonparametric tests. *P* values <0.05 were considered statistically significant.

## 3. Results

### 3.1. SLBZS Enhanced the Clinical Efficacy of Cefixime against Pneumonia in Children

The CONSORT flowchart of the trial is presented in Figure 1. There was no significant difference in age, gender, weight, and body mass index between the two groups (Table 1). Chest radiographs showed that both cefixime and cefixime + SLBZS treatments reduced the area of pulmonary inflammatory lesions relative to before treatment (Figure 2(a)). Additionally, the course of disease in the cefixime + SLBZS group was shorter than that in the cefixime group (Figure 2(b)). The total clinical efficacy rate of the cefixime and cefixime + SLBZS groups in treating pneumonia in children was 86.7% and 93.3%, respectively. Although the difference was at the limit of significance (*P*=0.335), the total clinical efficacy rate of the cefixime + SLBZS group was higher than that of the cefixime group (Table 2). Thus, treating pneumonia in children with cefixime + SLBZS was more effective than with cefixime alone. No obvious adverse reactions were observed, including diarrhea, nausea, aches, rashes, dizziness, and abnormal liver and kidney function.

The article "Shen-Ling-Bai-Zhu-San Enhances the Antipneumonia Effect of Cefixime in Children by Ameliorating Gut Microflora, Inflammation, and Immune Response" was retracted in 2023. Reasons: signs of a paper mill; suspected computer-generated content; unreliable results or conclusions; concerns about the data.

### 3.2. SLBZS Enhanced the Effects of Cefixime on WBC, Neutrophil, Lymphocyte Counts, and NLR

The blood cell analysis revealed that both cefixime and cefixime + SLBZS treatments decreased WBC and neutrophil counts and NLR relative to those prior treatments, indicating that cefixime + SLBZS treatment was more effective in reducing these cell counts (Figure 3). Both treatments increased the lymphocyte count in blood of children with pneumonia compared with before treatment. Cefixime + SLBZS was more effective than cefixime alone (Figure 3).

### 3.3. SLBZS Enhanced Cefixime Effect on Inflammatory Cytokine Levels

Both cefixime and cefixime + SLBZS treatments decreased the CRP, PCT, IFN-*γ*, TNF-*α*, IL-1*β*, IL-6, and IL-8 levels and increased IL-10 levels in serum of children with pneumonia. However, cefixime + SLBZS treatment was more effective than cefixime treatment (Figure 4).

### 3.4. SLBZS Enhanced Effects of Cefixime on Gut Microbiota

The gut microbiota culture results showed that cefixime and cefixime + SLBZS treatments decreased *Enterobacter*, *Enterococcus*, *Bacteroides*, and *Fusobacterium* counts in children with pneumonia. In addition, compared with cefixime, cefixime + SLBZS reduced the count of the four bacterial strains to levels closer to normal in children with pneumonia (Figure 5). Cefixime treatment decreased *Bifidobacterium* and *Lactobacillus* counts in the gut of children with pneumonia, whereas cefixime + SLBZS treatment increased *Bifidobacterium* and *Lactobacillus* counts to levels close to normal (Figure 5).

## 4. Discussion

Cefixime is frequently used as the initial antibiotic treatment prescribed for children with pneumonia. However, the decreasing susceptibility of respiratory pathogens to antibacterial agents has raised concerns over the reduced efficacy of currently available antibiotics [15]. SLBZS and cefixime treatments had the same result on *S. pneumoniae-*induced pneumonia mice, providing a new drug for treating pneumonia [14]. Therefore, we continued to investigate whether SLBZS could enhance the efficacy of cefixime in children with pneumonia. In the present study, we found that the total clinical efficacy rate of cefixime + SLBZS against pneumonia in children was higher than that of cefixime alone. Moreover, cefixime + SLBZS shortened the course of pneumonia in children. These results suggest that SLBZS could enhance the clinical efficacy of cefixime in children with this disease.

The article "Shen-Ling-Bai-Zhu-San Enhances the Antipneumonia Effect of Cefixime in Children by Ameliorating Gut Microflora, Inflammation, and Immune Response" was retracted in 2023. Reasons: signs of a paper mill; suspected computer-generated content; unreliable results or conclusions; concerns about the data.

Infection with pneumonia can cause increases in neutrophils, leukocytes, and NLR and decreases in lymphocytes in routine blood examinations [16]. Neutrophils, leukocytes, and NLR have a significant positive correlation. In contrast, lymphocytes significantly correlate with the pneumonia severity index, acting as a predictor for community-acquired pneumonia in healthy individuals [17]. Liang et al. reported similar findings in patients with severe pneumonia in a comparison between groups of nonsurvivors and survivors, which was consistent with the present study [18]. Furthermore, NLR was found to be a high-risk factor for 30-day mortality in patients with community-acquired pneumonia [19]. In addition, high neutrophils and NLR were associated with a higher risk of 90-day mortality [20]. Both cefixime and cefixime + SLBZS treatments reversed the above blood parameters in children with pneumonia. However, cefixime + SLBZS treatment was more effective than cefixime treatment alone.

Pneumonia promotes the secretion of inflammatory cytokines. PCT and CRP levels are increased during inflammatory disorders, providing useful serum markers for predicting pneumonia severity [21]. Thus, PCT may be a reliable biomarker for diagnosing hospital-acquired pneumonia in children [22]. Additionally, proinflammatory cytokines increase during pneumonia, whereas the level of IL-10, an anti-inflammatory cytokine that can oppose excessive inflammatory responses and reduce body injury, is decreased [23]. In a pneumonia mouse model, the expression of IL-1*β*, IL-6, IL-8, and TNF-*α* were enhanced, while IL-10 expression was reduced. The expression trend of the above inflammatory factors can be reversed after treatment [24, 25]. Similarly, in the present study, CRP, PCT, IFN-*γ*, TNF-*α*, IL-1*β*, IL-6, and IL-8 secretion increased, and IL-10 secretion decreased in children with pneumonia. Cefixime treatment inhibited CRP, PCT, IFN-*γ*, TNF-*α*, IL-1*β*, IL-6, and IL-8 secretion and increased IL-10 secretion, suggesting that cefixime treatment ameliorates symptoms of pneumonia in children by regulating inflammatory cytokine secretion. It has been shown that SLBZS treatment reduces inflammation to reverse nonalcoholic steatohepatitis progression [26]. Additionally, by decreasing IL-1*β* and TNF-*α* levels and increasing IL-10 levels, SLBZS treatment hinders inflammatory bowel disease development [27]. Similar to these results, cefixime + SLBZS treatment was more effective than cefixime treatment in suppressing CRP, PCT, IFN-*γ*, TNF-*α*, IL-1*β*, IL-6, and IL-8 secretion as well as promoting IL-10 secretion in children with pneumonia. This suggests that SLBZS enhances cefixime efficacy in regulating inflammatory cytokine secretion.

The article "Shen-Ling-Bai-Zhu-San Enhances the Antipneumonia Effect of Cefixime in Children by Ameliorating Gut Microflora, Inflammation, and Immune Response" was retracted in 2023. Reasons: signs of a paper mill; suspected computer-generated content; unreliable results or conclusions; concerns about the data.

A microbial imbalance in specific tissues is associated with disease development. The gut microbiota plays a protective role in host defense against pneumococcal pneumonia [12]. *Enterobacter, Enterococcus*, *Bacteroides*, and *Fusobacterium* are common causes of nosocomial pneumonia and also lead to drug resistance [28–31]. *Bifidobacterium* is among the dominant genera in the gut and has important effects on gut microbiota development during early and subsequent infant physiology and health [32]. There is ample evidence that *Bifidobacterium* and *Lactobacillus* supplementation positively affect the protection of the human gut from different intestinal infections. These microbes are associated with the production of beneficial metabolites [33, 34]. *Enterococcus* counts in patients with severe pneumonia were observed to be higher, while *Bifidobacterium* counts were lower than those in healthy people [35]. *Bifidobacterium longum*, *Lactobacillus bulgaricus,* and other probiotic treatments may be effective in preventing ventilator-associated pneumonia [36]. *Lactobacillus* and *Bifidobacterium* are probiotics that may effectively reduce the risk of antibiotic-associated diarrhea in hospitalized children with pneumonia [37]. However, cefixime treatment considerably reduces gut microbiota [38]. Similar to these findings, our results revealed that *Enterobacter, Enterococcus*, *Bacteroides*, and *Fusobacterium* counts were increased, whereas *Lactobacillus* and *Bifidobacterium* counts were decreased in children with pneumonia. Cefixime treatment decreases gut microbiota abundance, as seen in our previous study, where cefixime treatment decreased gut microbiota abundance in a *Streptococcus pneumoniae*-induced pneumonia murine model [14, 39]. The present study revealed that cefixime treatment could decrease microbial counts, suggesting that cefixime treatment had a broad-spectrum sterilization effect on microbiota, including *Lactobacillus* and *Bifidobacterium*. SLBZS treatment can ameliorate antibiotic drug-associated diarrhea by inducing structural changes in the gut microbiome [40]. SLBZS treatment reversed gut dysbiosis in functional dyspepsia rats as evidenced by reduced functional dyspepsia biomarkers, including *Prevotella*, *Mucispirillum*, and *Akkermansia* enrichment of SCFA-producing bacteria, such as *Adlercreutzia* and *Clostridium*, and sulfate-reducing bacteria, *Desulfovibrio* [9]. The present study also revealed that cefixime + SLBZS treatment could decrease *Enterobacter*, *Enterococcus*, *Bacteroides*, and *Fusobacterium* counts and increase *Bifidobacterium* and *Lactobacillus* counts in the gut of children with pneumonia. Thus, SLBZS might enhance the antipneumonia effect of cefixime in children with pneumonia by regulating the distribution and abundance of gut microbiota. The gut microbiota significantly correlates with neutrophils, leukocytes, NLR, lymphocytes, and inflammation. The lower NLR reflects a greater diversity of gut microbiota [41]. Abnormal intestinal bacterial secretions can activate neutrophils, leukocytes, and lymphocytes to regulate the secretion of inflammatory factors [42–45]. However, our results indicate whether intestinal flora, inflammation, and immune function are in an upstream and downstream regulatory relationship or a parallel relationship during treatment with SLBZS.

The article "Shen-Ling-Bai-Zhu-San Enhances the Antipneumonia Effect of Cefixime in Children by Ameliorating Gut Microflora, Inflammation, and Immune Response" was retracted in 2023. Reasons: signs of a paper mill; suspected computer-generated content; unreliable results or conclusions; concerns about the data.

## 5. Conclusions

SLBZS enhanced the clinical efficacy of cefixime in children with pneumonia by ameliorating gut microbiota, inflammation, and immune response. Thus, SLBZS combined with cefixime might be a potential treatment for pneumonia in children.

## Figures and Tables

**Figure 1:** CONSORT flowchart.

**Figure 2:** Effects of cefixime and cefixime + Shen-Ling-Bai-Zhu-San (SLBZS) treatments on pulmonary inflammatory lesion area and disease course in children with pneumonia. (a) The area of pulmonary inflammatory lesions after cefixime and cefixime + SLBZS treatments assessed using chest radiographs. (b) Disease course after cefixime and cefixime + SLBZS treatments (*n* = 30; ^*∗*^*P* < 0.05). Differences were analyzed using Student's *t*-test.

**Figure 3:** Effect of cefixime and cefixime + Shen-Ling-Bai-Zhu-San (SLBZS) treatments on white blood cell (WBC), neutrophil, lymphocyte counts, neutrophil-lymphocyte ratio (NLR), C-reactive protein (CRP), and procalcitonin (PCT) in blood of children with pneumonia (*n* = 30; ^*∗*^*P* < 0.05 vs. the normal group; ^#^*P* < 0.05, after vs. before cefixime treatment groups and after vs. before cefixime + SLBZS treatment group; and *P* < 0.05, after cefixime treatment groups vs. after cefixime + SLBZS treatment group). Differences between before and after treatment were analyzed using a paired *t*-test. ANOVA was used to compare five groups, followed by Tukey's post hoc test.

**Figure 4:** Interferon (IFN)-*γ*, tumor necrosis factor (TNF)-*α*, interleukin (IL)-1*β*, IL-6, IL-8, and IL-10 levels in serum of children with pneumonia measured using enzyme-linked immunosorbent assay (*n* = 30; ^*∗*^*P* < 0.05 vs. the normal group; ^#^*P* < 0.05 after vs. before cefixime treatment groups and after vs. before cefixime + SLBZS treatment group; and *P* < 0.05, after cefixime treatment groups vs. after cefixime + SLBZS treatment group). Differences between before and after treatment were analyzed using a paired *t*-test. ANOVA was used to compare five groups, followed by Tukey's post hoc test.

The article "Shen-Ling-Bai-Zhu-San Enhances the Antipneumonia Effect of Cefixime in Children by Ameliorating Gut Microflora, Inflammation, and Immune Response" was retracted in 2023. Reasons: signs of a paper mill; suspected computer-generated content; unreliable results or conclusions; concerns about the data.

**Figure 5:** Effects of cefixime and cefixime + Shen-Ling-Bai-Zhu-San (SLBZS) treatments on *Enterobacter*, *Enterococcus*, *Bacteroides*, *Bifidobacterium*, *Lactobacillus*, and *Fusobacterium* counts in the feces of children with pneumonia. The counts were measured by qPCR (*n* = 30; ^*∗*^*P* < 0.05 vs. the normal group; ^#^*P* < 0.05 after vs. before cefixime treatment groups and after vs. before cefixime + SLBZS treatment group; and *P* < 0.05, after cefixime treatment groups vs. after cefixime + SLBZS treatment group). Differences between before and after treatment were analyzed using a paired *t*-test. ANOVA was used to compare five groups, followed by Tukey's post hoc test.

**Table 1:** Baseline characteristics of the participants.

Characteristics	Cefixime group (*n* = 30)	Cefixime + SLBZS group (*n* = 30)
Age	6 (4, 7)	5 (4, 6.3)
Gender (male)	18 (60%)	16 (53.3%)
Weight	21.3 (18.73, 27.8)	20.7 (16.42, 25.50)
Body mass index	15.85 (14.78, 16.93)	15.95 (14.88, 16.73)

**Table 2:** Comparison of clinical efficacy between the two groups (cases (%)).

Groups	*n*	Obvious effective	Effective	Invalid	Total effective rate (%)
Cefixime group	30	12 (40.0%)	14 (46.7%)	4 (13.3%)	26 (86.7%)
Cefixime + SLBZS group	30	15 (50.0%)	13 (43.3%)	2 (6.7%)	28 (93.3%)

## Data Availability

The data used to support the findings of this study are included within the article.

## Abbreviations

SLBZS: Shen-Ling-Bai-Zhu-San
WBC: White blood cell
CRP: C-reactive protein
PCT: Procalcitonin
IFN-*γ*: Interferon-*γ*
TNF-*α*: Tumor necrosis factor-*α*
IL: Interleukin
ELISA: Enzyme-linked immunosorbent assay
CFUs: Colony-forming units.
